# Predictive significance of *TMRPSS2*-*ERG* fusion in prostate cancer: a meta-analysis

**DOI:** 10.1186/s12935-018-0672-2

**Published:** 2018-11-12

**Authors:** Chunjiao Song, Huan Chen

**Affiliations:** 1 Medical Research Center, Shaoxing People’s Hospital (Shaoxing Hospital, Zhejiang University School of Medicine), No. 568 Zhongxing Bei Road, Shaoxing, 312000 Zhejiang People’s Republic of China; 2 Zhejiang Institute of Microbiology (Key Laboratory of Microorganism Technology and Bioinformatics Research of Zhejiang Province), Hangzhou, Zhejiang China

**Keywords:** *TMPRSS2*-*ERG*, Fusion gene, Prostate cancer, Meta-analysis

## Abstract

**Background:**

Prostate cancer is a major malignancy in males. *TMPRSS2*-*ERG* is a high-frequency fusion gene expressed in prostate cancer and plays a vital role in carcinogenesis. Recent studies showed that *TMPRSS2*-*ERG* is a potential predictive biomarker for prostate cancer. However, the predictive value of *TMPRSS2*-*ERG* fusion is yet unclear.

**Methods:**

A total of 76 relevant articles, published from 2015 to 2017, were obtained from PubMed, Web of Science, EMBASE, Scopus, the Cochrane Library, and CNKI databases to investigate the predictive significance of *TMPRSS2*-*ERG* fusion in prostate cancer. Pooled odds ratio (ORs) with 95% confidence intervals (CIs) were calculated to estimate the correlation between *TMPRSS2*-*ERG* fusion gene and tumor features.

**Results:**

The pooled or stratified analysis showed that the *TMPRSS2*-*ERG* fusion gene had a highly predictive potential. First, *TMPRSS2*-*ERG* fusion was associated with T-stage at diagnosis (T3–4 vs. T1–2 OR: 1.40; 95% CI 1.33–1.48) and metastasis (M1 vs. M0 OR: 1.35; 95% CI 1.02–1.78) but not with biochemical recurrence or prostate cancer-specific mortality. Furthermore, the subgroup analysis found that the *TMPRSS2*-*ERG* fusion gene was correlated with Gleason (G) scores, and the fusion was common in prostate cancer with G ≤ 7. Additionally, the meta-analysis demonstrated that the fusion was likely to occur in young patients (> 65 vs. ≤ 65 OR: 0.68; 95% CI 0.52–0.89), in patients with high PSA levels (> 10 vs. ≤ 10 OR: 1.30; 95% CI 1.21–1.38), and in patients with peripheral involvement (positive vs. negative OR: 1.17; 95% CI 1.08–1.28), while not associated with tumor volume. Finally, the subgroup analysis of different fusion types demonstrated that the deletion-type fusion was significantly associated with the malignant degree of prostate cancer (pooled OR: 5.67; 95% CI 2.85–11.28). Moreover, the deletion-type was common in Africa patients, followed by Caucasian patients, and no significant difference was observed in the incidence of different fusion types in the Asian population.

**Conclusions:**

The meta-analysis findings suggested that the *TMPRSS2*-*ERG* fusion gene might be a predictive marker for prostate cancer patients, and might be valuable for assessing the characteristics of prostate cancer for individualized treatment and prognosis evaluation.

**Electronic supplementary material:**

The online version of this article (10.1186/s12935-018-0672-2) contains supplementary material, which is available to authorized users.

## Background

Prostate cancer (PCa) is the most common non-skin cancer and a leading male malignancy worldwide. In 2017, 161,360 new cases were recorded, and 26,730 patients died of PCa in the USA [1]. According to the recent data of the National Center for Cancer, PCa has the highest rate of occurrence of tumors in the urinary system since 2008 in China [2]. The morbidity rate was ranked sixth, while the mortality rate was ninth in all the male malignant tumors [2]. PCa is initially limited to the prostate and curable by a variety of therapeutic methods. However, about 23–40% of these patients with PCa would develop into CRPC (castration-resistant prostate cancer) or mCRPC (metastatic castration-resistant prostate cancer) after the primary treatment of PCa, which is usually untreatable [3]. Metastatic PCa cells tend to metastasize to the liver, lung, bone, other visceral organs, as well as to the skin, leading to the death of the patient [4].

In the 1990s, the screening for PSA (prostate-specific antigen), widely used in clinical practice, led to a significant increase in PCa cases [5]. However, the PSA level was not specific for PCa and may fluctuate due to other prostatic diseases: inflammation, infection, or hyperplasia. Therefore, the diagnostic specificity of PSA was not high, which might lead to false-positives and overtreatment [6]. Moreover, 15% of the males with low PSA levels would progress towards PCa [6]. As a result, the US Preventive Services Task Force recommended that PSA levels were not detected routinely, and PSA tests were only used for high-risk populations [7]. In addition, the diagnostic sensitivity of prostate needle biopsy was also low, with about 40% of the diagnostic results being false-negative, and only 2% of the PCa tissues could be sampled [6, 8]. Thus, specific and precise biomarkers to accurately detect PCa and distinguish the different stages of PCa are yet to be elucidated.

In 2005, Tomlin et al. reported the first gene fusion of *TMPRSS2* (transmembrane protease, serine 2) gene and *ERG* (ETS (erythroblast transformation-specific)-related gene), the most common form of PCa-specific fusions [9]. Since then, the *TMPRSS2*-*ERG* fusion is the hotspot of the related studies on PCa. *TMPRSS2*-*ERG* fusion gene is specifically expressed in PCa, involving the *TMPRSS2* gene regulated by androgen and the oncogene *ERG* that is a member of the ETS family of transcription factors. The fusion frequency of *TMPRSS2*-*ERG* was about 50% in Caucasian Americans (CA), 31% in African Americans (AA) [10], and 18.5% in Asians [11]. The fusion gene may result in a high expression of *ERG* by driving the androgen reaction element (ARE) of the *TMPRSS2* gene [12], which plays a critical role in the regulation of cell growth, differentiation, and apoptosis [13]. This phenomenon indicates that *TMPRSS2*-*ERG* fusion may be a driver of PCa progression by affecting a series of downstream oncogenic effects. Thus, the *TMPRSS2*–*ERG* gene is considered to be an early event in the development of PCa. Furthermore, *TMPRSS2*-*ERG* gene fusion can be generated by chromosomal translocation or interstitial deletion [14, 15]. The frequency of translocation, deletion, and concurrence was 61.9%, 38.1%, and 0% in CA patients, while 20%, 60%, and 20% in AA cases, respectively [10].

*TMPRSS2*-*ERG* is an attractive biomarker as it can be accurately detected from various biological samples by several methods. For example, the gene rearrangement can be determined using fluorescence in situ hybridization (FISH) [9, 15], the expression level can be measured by polymerase chain reaction (PCR) [9], and the overexpression of ERG can be detected using immunohistochemistry (IHC) [16]. Moreover, a noninvasive diagnostic strategy was developed to clinically detect the fusion transcripts in patients’ urine samples [17, 18]. However, some studies on *TMPRSS2*-*ERG* fusion as the predictive biomarker for PCa based on different patient cohorts, detection methods, or data analysis platforms are yet controversial. Therefore, we systematically performed the meta-analysis to clarify the predictive accuracy of *TMPRSS2*-*ERG* in clinical PCa specimens.

## Materials and methods

### Search strategy

The meta-analysis was performed according to the standard guidelines for tumor biomarker studies. We searched PubMed, Web of Science, Embase, Scopus, the Cochrane Library, and Chinese National Knowledge Infrastructure (CNKI) databases to retrieve the relevant articles, published between 2005 and 2017, on the predictive value of *TMPRSS2-ERG* fusion gene in patients with PCa. The search strategy was a combination of Medical Subject Headings (MeSH) terminology and keywords as follows: (“prostate cancer” or “prostate carcinoma” or “prostate neoplasm” or “prostate tumor/tumor”) and (“TMPRSS2-ERG” or “TMPRSS2-ETS”) and (“marker” or “biomarker”). The selected articles were viewed carefully, and the reference lists were also screened to identify other eligible publications (Fig. 1). The literature search was completed on Dec 20, 2017.

**Fig. 1:** Flowchart of study selection process in this meta-analysis

### Inclusion and exclusion criteria

According to the inclusion and exclusion criteria, the abstracts and the full texts of the relevant articles were screened for eligibility. A total of 197 primary studies and 43 additional records from reviews or meta-analysis were retrieved, and 76 publications were included in this meta-analysis (Fig. 1).

The studies selected for the meta-analysis were required to fulfill the following inclusion criteria: (1) *TMPRSS2*-*ERG* fusion status was identified. (2) All cases involved in these studies should have been verified by gold standard test (pathological confirmation for the diagnosis of PCa). (3) Sufficient data were reported to calculate the odds ratio (ORs) and the 95% confidence intervals (CIs). (4) The level of *TMPRSS2*-*ERG* was assessed in prostatic tissues or blood or urine samples.

The exclusion criteria for the study were as follows: (1) The studies were not original articles, such as reviews, letters, commentaries, erratums, and meta-analysis. (2) Data for *TMPRSS2*-*ERG* fusion gene were not sufficient for extraction. (3) Non-English or non-Chinese language. (4) Data were obtained from non-human samples or human cell lines. (5) Duplicate records.

### Data extraction

Data were extracted from all eligible studies using a standardized form to evaluate the association between the *TMPRSS2*-*ERG* fusion gene and PCa outcomes (tumor stage, Gleason (G) score, biochemical recurrence, lethal PCa) and PCa clinical features (age at diagnosis, PSA level, tumor volume). In addition, the following information was collected: country, year of publication, the first author, patients’ age, PSA level, tumor volume, the number of samples, detection strategy, and the diagnostic data (negative, positive, translocation-type, and deletion-type). Moreover, some articles reported the results of multiple subgroups, and hence, we extracted the data of each subgroup as an independent cohort to perform the meta-analysis.

### Quality assessment

The quality of all included studies was assessed using Revman 5.3 software (Cochrane, London, UK). This software can be utilized to draw funnel plots to represent the publication bias, and these biased studies are distributed outside the edges. Simultaneously, the heterogeneity of the publications can be found by combining the I^2^ value (the inconsistency index) and P-value (Chi squared). If the I^2^ value is > 50% and the P-value is < 0.1, heterogeneity was ascribed in this analysis. Conversely, the heterogeneity of the articles was extremely low. Furthermore, to avoid the effects of heterogeneity, we performed subgroup analyses by classifying the included studies into several subgroups based on the methods, patients’ races, and sample types.

### Statistical analysis

The statistical analyses for the meta-analysis were performed using Revman 5.3 to calculate the overall predictive accuracy. Pooled ORs with 95% CIs and forest plots were used to assess the predictive role of *TMPRSS2*-*ERG* fusion gene in various stages of PCas. All P-values were two-tailed and P < 0.05 was considered to be statistically significant unless otherwise specified.

## Results

### Characteristics of included studies

According to our search strategy, a total of 197 primary studies and 43 additional studies were retrieved from PubMed, Web of Science, Embase, Scopus, the Cochrane Library, and CNKI databases. Figure 1 summarized the selection process for the systematic literature search. Finally, a total of 76 studies were included in this study after carefully reviewing the abstracts and full texts, and 42,997 cases (34,219 localized PCa, 360 metastatic PCa, 256 CRPC, 167 HGPIN (high-grade prostate intraepithelial neoplasia), 255 BPH (benign prostate hyperplasia), and 7740 normal) were analyzed statistically based on different indices of the meta-analysis. Two studies were removed due to data duplication. Also, the following studies were excluded: review or meta-analysis or commentary (n = 23), studies belonging to basic research (n = 50), studies without sufficient relevant data (n = 84), methodological studies (n = 4), and non-English or non-Chinese articles (n = 1).

The primary characteristics of the 76 included studies were summarized in Additional file 1: Table S1 in the order of the published year and authors’ surname. The publication period of these studies ranged from 2005 to 2017. In addition, some studies could be divided into several parts because they included multiple research cohorts. The data from these records were collected from all over the world, including 18 countries or regions except Africa. The dominant race in 60 studies was Caucasian, while 17 studies were executed in Asia. The fusion status and the expression level of *TMPRSS2*-*ERG* were detected using FISH (n = 47), IHC (n = 21), qRT-PCR (n = 26), and transcription-mediated amplification (TMA) (n = 2) in prostate tissues (n = 72), while 1 study examined the blood samples and 5 studies utilized urine samples (Additional file 1: Table S1). In these studies, data from a total of 42,830 cases were available for the meta-analysis, with a minimum sample size of 19 and a maximum sample size of 11,152 patients. The diagnosis of patients with PCa was based on the pathological confirmation.

We calculated the pooled ORs and the 95% CIs to evaluate the association between *TMPRSS2*-*ERG* fusion and PCa outcomes: T-stage (T3–4 vs. T1–2), G (8–10 vs. 1–7), biochemical recurrence (positive vs. negative), and lethal PCa (positive vs. negative). Also, we assessed the association among age at diagnosis, PSA level, and tumor volume. Finally, we extracted the available data and performed subgroup analyses comparing the *TMPRSS2*-*ERG*-positive patients with deletion-type to other fusion types.

### *TMPRSS2*-*ERG* fusion and prostate cancer outcomes

#### Tumor stage

TNM (tumor node metastasis) is the staging of tumor in oncology, which was first presented by Pierre Denoix of France from 1943 to 1952. Then, American Joint Committee on Cancer (AJCC) and Union for International Cancer Control (UICC) gradually established the international staging criteria: (1) T (tumor) refers to the primary tumor lesion, with an increase in the tumor volume and the involved range of adjacent tissues, defined as T1–T4. (2) N (node) refers to the affected regional lymph nodes. When the lymph nodes are not affected, N0 is used. As the degree and scope of lymph node involvement is increased, N1–N3 are utilized. (3) M (metastasis) is defined as the tumor that is spread primarily through the blood channel; there is no distant metastasis represented by M0, and there are distant metastases in terms of M1.

The risk for the association between the *TMPRSS2*-*ERG* fusion and the PCa stages was estimated. In Fig. 2a, d, we found that *TMPRSS2*-*ERG* fusion was more common in the T3–4 stages of PCa than in the T1–2 after excluding the two studies with heterogeneity Petterson et al. [19] and Zhou et al. [20] (P < 0.01), and the pooled OR and 95% CI was 1.40 (1.33–1.48). However, no statistical difference was detected in the analysis of N (P = 0.26). Thus, it can be speculated that *TMPRSS2*-*ERG* fusion was not associated with the adjacent lymph nodes, irrespective of whether they were affected (Fig. 2b, e). Moreover, a significant difference was detected in the comparison between M1 and M0 (P = 0.04), the pooled OR and 95% CI was 1.35 (1.02–1.78), respectively. In the M1 cases with distant metastases, *TMRPSS2*-*ERG* fusion was frequent (Fig. 2c, f).

**Fig. 2:** Meta-analysis for prostate cancer outcomes. Forest plots show the pooled ORs and 95% CIs of *TMPRSS2*-*ERG* fusion gene with corresponding heterogeneity statistics. Squares and horizontal lines correspond to the study-specific ORs and 95% CIs; respectively. The area of the squares correlates with the weight of each enrolled study, and the diamonds represent the summary ORs and 95% CIs. Funnel plots are the assessment of potential publication bias. **a** Forest plot for the analysis of primary tumor; **b** forest plot for the analysis of adjacent lymph node; **c** forest plot for the analysis of metastasis; **d** funnel plot for primary tumor; (E) Funnel plot for adjacent lymph node; **f** funnel plot for metastasis; **g** forest plot for the analysis of biochemical recurrence; **h** forest plot for clinical recurrence; **i** forest plot for the analysis of prostate cancer-specific death; **j** funnel plot for the analysis of biochemical recurrence; **k** funnel plot for the analysis of potential publication bias of tumor-specific death

#### G score

We carried out the subgroup analyses on the *TMPRSS2*-*ERG* fusion gene in PCa with different G scores after excluding several studies, which might be the main source of heterogeneity. In the subgroup analysis classified by different detection methods (Fig. 3a, d), the data of FISH and IHC groups showed that *TMPRSS2*-*ERG* fusion was more frequent in G ≤ 7 PCa than in G > 7 (P < 0.01). Consequently, the P-value of RT-PCR group was 0.11, the pooled ORs and 95% CIs were 0.63 (0.52–0.75) in the FISH group, 0.80 (0.61–1.05) in the RT-PCR group, and 0.79 (0.68–0.91) in the IHC group, respectively. Moreover, the total P-value was < 0.01, and the total OR and 95% CI was 0.73 (0.66–0.81). The difference among FISH, RT-PCR, and IHC groups was not significant (P = 0.14, I^2^ = 49.9%). The race subgroup analysis showed that *TMPRSS2*-*ERG* fusion was common in G ≤ 7 PCa (Fig. 3b, e), irrespective of Caucasian PCa (P < 0.01) or in Asian PCa (P = 0.08). The pooled ORs and 95% CIs was 0.81 (0.72–0.90) in the Caucasian group and 0.74 (0.53–1.03) in the Asian group, respectively. The summarized P-value was < 0.01, and the total OR and 95% CI was 0.80 (0.72–0.89), and no difference was observed between the Caucasian and Asian groups (P = 0.65, I^2^ = 0%). Also, the subgroup analysis of different sample types indicated that *TMPRSS2*-*ERG* fusion was common in G ≤ 7 PCa [P < 0.01, OR 95% CI: 0.73 (0.66–0.80)] (Fig. 3c, f). Only one study utilized urine samples, and the OR and 95% CI was 1.82 (0.66–5.03), indicating that *TMPRSS2*-*ERG* fusion was common in G > 7 PCa. This phenomenon might be attributed to the malignant PCa shedding the tumor cells into urine that can be detected. In addition, after carefully reviewing the full-texts, we confirmed that heterogeneity was primarily caused by 6 studies: Demichelis et al. [21], Attard et al. [22], Hu et al. [23], Sun et al. [24], Kulda et al. [25], and Liu et al. [26].

**Fig. 3:** Subgroup analysis for the Gleason score of prostate cancer. Forest plots of subgroup analyses stratified by detected methods, ethnicities, and sample types show *TMRPSS2*-*ERG* fusion gene with corresponding heterogeneity statistics. Squares and horizontal lines correspond to study-specific ORs and 95% CIs; respectively. The area of the squares correlates with the weight of each enrolled study, and the diamonds represent the summary ORs and 95% CIs. Funnel plots represent the assessment of potential publication bias. The forest plots for **a** subgroup analysis stratified by detection methods, **b** subgroup analysis stratified by different races, **c** subgroup analysis stratified by sample types. The funnel plots for **d** subgroup analysis stratified by methods, **e** subgroup analysis stratified by races, **f** subgroup analysis stratified by sample types

#### Biochemical recurrence

After removing a highly heterogeneous study (Barwick et al. [27]), the result did not present any association between *TMPRSS2*-*ERG* fusion and biochemical recurrence (P = 0.37) as shown in Fig. 2g, j, and there was no correlation between the fusion status and clinical recurrence as shown in Fig. 2h (P = 0.43). Moreover, the meta-analysis included 2556 patients who were followed up for biochemical recurrence (697 events) and 510 cases for clinical recurrence (109 events).

#### Prostate cancer-specific death

As shown in Fig. 2i, k, the meta-analysis included 211 males who were deceased due to PCa and 1947 males with PCa survived. However, there was no statistically significant difference in males with *TMPRSS2*-*ERG* fusion-positive tumors as compared to those with negative fusion (P = 0.49), and the pooled OR was 1.11 (95% CI 0.82–1.50).

### Other clinical features

#### Age at diagnosis

Figure 4a, d demonstrated the pooled OR and 95% CI, which was calculated to assess the association between the fusion status and age at diagnosis. The integrated result suggested that *TMRPSS2*-*ERG* fusion was associated with age (P < 0.01), the pooled OR and 95% CI was 0.68 (0.52–0.89). The *TMPRSS2*-*ERG* fusion was common in young males with PCa (age ≤ 65 years), which was consistent with a previous study [28]. The intrinsic reason might be high levels of androgen in young patients that are likely to induce *TMPRSS2*-*ERG* fusion.

**Fig. 4:** Meta-analysis of the general clinical features for prostate cancer patients. Forest plots for **a** age at diagnosis, **b** serum PSA level, **c** tumor volume. Funnel plots for **d** age, **e** PSA; **f** forest plot for surgery margin involvement; **g** funnel plot for margin; **h** forest plot for perineural invasion

#### Serum PSA level

As shown in Fig. 4b, e, the pooled result implied that *TMPRSS2*-*ERG* fusion was associated with serum PSA level (P < 0.01). The positive fusion was detected frequently in the PCa patients with a high level of PSA (> 10 ng/mL), and the calculated OR and 95% CI was 1.30 (1.21–1.38). Among these included studies, Attard et al. [22] affected the result greatly, thereby indicating the high heterogeneity of the study.

#### Tumor volume

The detection of the fusion in urine was excluded using TMA method [29], and we found that *TMPRSS2*-*ERG* fusion was not associated with tumor size (P = 0.40) (Fig. 4c). However, this phenomenon might be attributed to the little data extracted from these studies, and hence, additional studies are essential to confirm the correlation between *TMPRSS2*-*ERG* fusion and PCa volume.

#### Margin invasion

We analyzed the correlation between *TMPRSS2*-*ERG* fusion status and surgical margins. In Fig. 4f, g, the fusion was correlated to the involvement of the surgical margin (P < 0.01), and the pooled OR and 95% CI was 1.17 (1.08–1.28). Consequently, *TMPRSS2*-*ERG* fusion was positive in patients with surgical margin invaded by tumor cells.

#### Perineural invasion

Furthermore, we also discussed whether the fusion was correlated to the invasion of peripheral nerves. The meta-analysis result showed that a negative association between the fusion status and perineural invasion (P = 0.06) (Fig. 4h), which might be due to the little data in the study. Thus, we speculated a slight statistical significance; *TMPRSS2*-*ERG* fusion was likely to be detected in the cases of peripheral nerve involvement.

### Deletion-type fusion and prostate cancer

Furthermore, we collected the data about the numbers of different fusion types in PCa tissues, including deletion-type fusion, translocation-type fusion, and amplification-type. In addition, the subgroup analyses were shown in Fig. 5. Since the fusion subtypes of *TMPRSS2*-*ERG* must be detected using FISH in tissue samples; the subgroup analyses mainly involved the race subgroup (Fig. 5a, c), and the results did not show any obvious difference (P = 0.66) with respect to the Asians. On the other hand, in the Caucasian and African groups, deletion-type fusion was common (P < 0.01). The pooled OR and 95% CI was 1.77 (1.50–2.09) in the Caucasian group, while only one study provided complete data available for analysis in the African group with OR and 95% CI 2.25 (0.63–7.97). The total P-value was < 0.01, while the total OR and 95% CI was 1.68 (1.43–1.97). The difference between the three groups was slightly significant (P = 0.07, I^2^ = 63.1%), and the results were not consistent with those from previous studies [10, 11]. Moreover, after the removal of highly heterogeneous studies, only 5 performed in Asian population were considered. Of these, only 1 study on the African patients was included, and 19 studies provided the complete data for analysis in the Caucasian population. Thus, the conclusion might be incomplete, necessitating additional investigations.

**Fig. 5:** The subgroup analysis assessed the association between *TMPRSS2*-*ERG* fusion subtypes and prostate cancer. Forest plots show the subgroup analyses of deletion-type fusion versus other fusion types. Squares and horizontal lines correspond to study-specific ORs and 95% CIs; respectively. The area of the squares correlates with the weight of each enrolled study, and the diamonds represent the summary ORs and 95% CIs. Funnel plots indicate the assessment of the potential publication bias. **a** forest plot for the subgroup analysis of different races; **b** funnel plot evaluating the heterogeneity for the subgroup analysis in different races; **c** forest plot for the subgroup analysis in metastatic PCa or CRPC; **d** funnel plot for the subgroup analysis in metastatic PCa or CRPC

Furthermore, the subgroup analyses elucidated the differences of *TMPRSS2*-*ERG* fusion types in metastatic PCa or CRPC groups (Fig. 5b, d). The meta-analysis results showed that the deletion-type fusion was common in metastatic PCa or CRPC (P < 0.01), and the pooled ORs and 95% CIs were 3.68 (1.43–9.48) and 9.41 (3.37–26.30), respectively. The summarized P-value was < 0.01, and the total OR and 95% CI was 5.67 (2.85–11.28) without a significant difference between metastatic PCa and CRPC groups (P = 0.19, I^2^ = 42.5%). Only limited data were available for the subgroup analysis to confirm the predictive value of different fusion types, and hence, further studies with large sample size studies are imperative.

## Discussion

Since *TMPRSS2*-*ERG* fusion was discovered in 2005, the specific fusion gene had been extensively studied as a potential predictive biomarker for PCa. However, the clinical value of *TMPRSS2*-*ERG* fusion is yet controversial because of different results as well as contrasting conclusions. Herein, we investigated the application value of *TMPRSS2*-*ERG* fusion for PCa by meta-analysis of all relevant included studies. The meta-analysis demonstrated that *ERG* overexpression or positive fusion status was associated with advanced pathological characteristics of PCa. This phenomenon was inconsistent with the reports, wherein the frequency of *TMPRSS2*-*ERG* fusion was shown to be 50% in in situ carcinoma and decreased in malignant PCa [30]. Moreover, some studies reported a positive association between *TMPRSS2*-*ERG* fusion and clinicopathological features [15, 21, 22, 31–33], while other studies put forth a negative association [34–44]. In the systematic meta-analysis, our results demonstrated that *TMPRSS2*-*ERG* fusion was significantly associated with T-stages, metastasis, and G scores in PCa patients. Moreover, the fusion gene was common in young patients, in patients with high PSA levels, and in cases with peripheral involvement. The prevalence of the fusion was 52.4% in Caucasian cohorts, 36.3% in African cohorts, and 47.5% in Asian cohorts, which was different from the reports that the frequency of *TMPRSS2*-*ERG* fusion was about 20% in Asia [11]. The current meta-analysis did not find any association between *ERG* overexpression or *TMPRSS2*-*ERG*-positive fusion and the risk of tumor recurrence; a similar result was found with PCa-specific death that was consistent with a previous meta-analysis [19]. The study also yielded a similarly negative result for tumor volume, while the study by Schaefer reported that *ERG* overexpression was inversely correlated with the tumor size [45]. In addition, the subgroup analyses for the frequency of deletion-type of *TMPRSS2*-*ERG* fusion in different races and metastatic PCa or CRPC were conducted. Compared to the translocation or other patterns, the prognosis of PCa patients with deletion-type fusion was poor. Since the 2.8 Mb region was located between *TMPRSS2* and *ERG* genes on chromosome 21 was lost in the deletion-type fusion, it was speculated that this region might contain critical tumor suppressors [46]. The current meta-analysis results exhibited that the incidence of deletion-type fusion was significantly higher in malignant PCa. Additionally, the deletion-type fusion was most common in African patients, followed by Caucasians, while no statistical difference was noted between deletion-type fusion and translocation-type fusion in Asian populations. However, limited data were collected from a limited number of appropriate studies, and hence, additional standardized data were required from large-sample multicenter trials to substantiate the current findings.

Notably, the high heterogeneity in these included studies was used to estimate the predictive accuracy of *TMPRSS2*-*ERG* fusion. The difference might be induced by the detection techniques, race of the study cohorts, the sample types, and the limited number of events in these studies. Among them, the results were highly heterogeneous in urine detections, which might be attributed to distinct urine components. Thus, the suspected negative cases should be examined multiple times to avoid misdiagnosis in the urine tests. Furthermore, subgroup analyses evaluated the diagnostic value of *TMPRSS2*-*ERG* fusion based on the different detection methods (FISH, RT-PCR, or IHC). In order to reduce the effects of the patients’ ethnic groups with different genetic backgrounds, we classified the included studies into Caucasian, African, and Asian groups. Simultaneously, we also categorized the enrolled studies into three groups depending on the sample types (tissue, serum, or urine) to conduct subgroup analyses. The detection of the fusion gene in the tissues has been widely accepted by medical staff. However, the detection in serum or urine samples was attractive because it was noninvasive and convenient, which could be used to dynamically monitor the progress of the disease and the therapeutic effect at any time in the case of PCa patients.

Nevertheless, the meta-analysis has many merits. First, the current data from were recorded from the literature in strict accordance with inclusion criteria. Second, the qualities of the included literature were satisfactorily assessed by Revman 5.3 software. Third, we performed the subgroup analyses to effectively avoid the effects of heterogeneity and to explore the scope of application for *TMPRSS2*-*ERG* fusion as a predictive biomarker for PCa.

The meta-analysis also had some shortcomings. First, *TMPRSS2*-*ERG* positive fusion is only a subtype of PCa, and it cannot identify approximately 50% of the patients, which limits its clinical application. When the result of fusion gene detection is negative, the risk of PCa cannot be excluded. On the other hand, both *TMPRSS2* and *ERG* genes have multiple fusion partners, and these fusion variants are also associated with PCa outcomes [32, 47, 48]. In the present meta-analysis, we evaluated the clinical value of *TMPRSS2*-*ERG* fusion at a maximal frequency in PCa. Strikingly, *TMPRSS2*-*ERG* fusion detection may be limited as the first-line detection, but due to the high specificity for PCa, confirming the diagnosis and determining the subtype for personalized treatment is essential.

Second, some results of the meta-analysis were obtained from the limited available data after removing the several records because of high heterogeneity; for example, the analyses on metastatic PCa and CRPC, the analyses on clinical recurrence and lethal PCa, and the analyses on tumor volume and peripheral involvement. Therefore, multicenter large-scale studies with high-quality are essential to confirm the current findings.

Third, some results did not exhibit a statistical significance after data consolidation and stratification analysis. While some were indistinguishable, others did not have sufficient data for analysis.

Finally, as there was no uniform cut-off value for *ERG* expression level measured by RT-PCR or IHC, the evaluation of TMPRSS2-ERG fusion as a PCa biomarker was not accurate. The ERG score was utilized for further calculated based on the equation: TMPRSS2-ERG/PSA × 100,000. *TMPRSS2*-*ERG* score was also assessed as a dichotomous variable that *TMPRSS2*-*ERG*-positive fusion was defined as copies > 10. Both RT-PCR and IHC were indirect methods and could not evaluate the fusion status unlike FISH, which was a well-standardized and expensive method requiring only a small amount of tumor tissue. It could directly determine the fusion state and easily identify the other fusion types of *TMPRSS2*-*ERG* transcripts. However, FISH was only used in surgical tissues, and body fluid-based detection was not reported.

In summary, the application value of *TMPRSS2*-*ERG* fusion as a predictive factor for PCa was not elucidated, requiring additional data for substantiation of the hypothesis. In addition, the meta-analysis revealed that future studies should be more designed such as to consider the further application of the data. Finally, because *TMPRSS2*-*ERG* fusion occurred only in about 50% of the PCas [37], the combination of multiplex gene predictors’ detection essentially replaced a single *TMPRSS2*-*ERG* to improve the predictive accuracy.

## Conclusions

The meta-analysis carried out an omnidirectional analysis on the correlation between *TMPRSS2*-*ERG* fusion gene with various clinical characteristics of PCa. The *TMPRSS2*-*ERG* fusion was associated with stages, metastasis, and Gleason scores of PCa, while it was not associated with the involvement of the lymph node. In addition, the fusion status was not associated with tumor volume, PCa recurrence, or PCa specific death. Also, we found that *TMPRSS2*-*ERG* fusion was frequent in young patients, in patients with high PSA levels, and in patients with perineural involvement. Finally, the analysis of ratios of different fusion types in PCa cases demonstrated that the deletion-type fusion had the highest proportion in the black men with PCa, followed by white, and in the Asian population, no difference was observed among the fusion subtypes. Consecutively, the deletion-type fusion was common in the malignant mCRPC, which might be correlated to the loss of tumor suppressor genes located between *TMPRSS2* and *ERG* genes.

## Additional file

**Additional file 1: Table S1.** The main characteristics of the included studies.

## Abbreviations

AA: African American
AJCC: American Joint Committee on Cancer
ARE: androgen reaction element
BPH: benign prostate hyperplasia
CA: Caucasian American
CIs: confidence intervals
CNKI: Chinese National Knowledge Infrastructure
CRPC: castration resistant prostate cancer
DASL: cDNA-mediated, annealing, selection, extension and ligation
*ERG*: ETS-related gene
*ETS*: erythroblast transformation-specific
FISH: fluorescence in situ hybridization
HGPIN: High Grade Prostate Intraepithelial Neoplasia
IHC: immunohistochemistry
MeSH: Medical Subject Headings
ORs: odd ratios
PCa: prostate cancer
PCR: polymerase chain reaction
PSA: prostate-specific antigen
qRT-PCR: quantitative real-time polymerase chain reaction
SPSS: Statistical Product and Service Solutions
TMA: transcription mediated amplification
TMPRSS2: transmembrane protease, serine 2
TNM: tumor node metastasis
UICC: Union for International Cancer Control
